This article has been retracted.

# Neuroprotective Effects of Probiotic-Supplemented Diet on Cognitive Behavior of 3xTg-AD Mice

**DOI:** 10.1155/2022/4602428

**Published:** 2022-01-05

**Authors:** Chenxi Tan, Yang Liu, Huiyi Zhang, Cihan Di, Dechao Xu, Chunming Liang, Ningning Zhang, Bing Han, Weiya Lang

**Affiliations:** ^1^Ward 5, Department of Neurology, The Second Affiliated Hospital of Qiqihar Medical University, Qiqihar 161000, China; ^2^Ward 1, Department of Neurology, The Second Affiliated Hospital of Qiqihar Medical University, Qiqihar 161000, China; ^3^Department of Pathology, School of Basic Medicine, Qiqihar Medical University, Qiqihar 161000, China; ^4^Department of Rehabilitation, The Second Affiliated Hospital of Qiqihar Medical University, Qiqihar 161000, China; ^5^Department of Tissue Culture, School of Basic Medicine, Qiqihar Medical University, Qiqihar 161000, China

## Abstract

Alzheimer's disease (AD) is recognized as one of the most common types of senile dementia. AD patients first suffer memory loss for recent events (short-term memory impairment). As the disease progresses, they are deprived of self-awareness. This study aims to explore the effects of a probiotic-supplemented diet on the cognitive behaviors and pathological features of mouse models of Alzheimer's disease (AD). Mice in the control group and the 3xTg-AD group were fed a regular diet and a probiotic-supplemented diet, respectively, for 20 weeks. Behavioral experiments like Morris's water maze and Y maze were conducted. Then, feces of mice were collected for 16S sRNA gene sequencing for microorganisms. In the end, soluble and insoluble A*β*40 and A*β*42 in the hippocampus and cortex of mice in each group were quantitatively analyzed with a double-antibody Sandwich ELISA. The expression levels of tau protein and gliocyte in the hippocampus and cortex were detected using the Western Blot method. The result of the Morris water maze experiment indicated that, in the place navigation test, the mice in the 3xTg-AD group experienced a significant decline in the learning ability and a longer escape latency and in the space exploration test, the swimming time of mice in the 3xTg-AD group in the target quadrant decreased and after being treated with the probiotic diet, mice in the 3xTg-AD group had improved learning and memory ability. The result of Y maze showed that the probiotic diet can improve the spontaneous alternation accuracy of mice in the 3xTg-AD group. The result of 16s rRNA gene sequencing showed that, compared with mice in the WT group, those in the 3xTg-AD group experienced a change in the intestinal flora. The Western Blot result displayed a decreased expression level of tau (pS202) (*P* < 0.05) and decreased expression levels of Iba-1 and GFAP (*P* < 0.05). The result of the ELISA experiment showed decreased levels of soluble and insoluble A*β*40 and A*β*42 in 3xTg-AD mice (*P* < 0.05). In conclusion, a probiotic diet can prevent and treat AD by improving the intestinal flora of 3xTg-AD.

## 1. Introduction

Alzheimer's disease (AD) is recognized as one of the most common types of senile dementia [1]. AD patients first suffer memory loss for recent events (short-term memory impairment). As the disease progresses, they are deprived of self-awareness [2]. Early onset of AD, old age, low education level, and some poor physical conditions affect the prevalence rate of the disease and the severity of cognitive disorder [3]. Alteration of intestinal microflora [4], cognitive disorder [5], and neuroinflammation [6] were reported to be associated with many central nervous systems (CNS) neurodegenerative diseases including AD. Experimental evidence showed that a change in the micronutrients is also a hazardous factor of AD [7]. At present, there is no definite therapy for AD. The therapies available can protect cognition and memory and delay the loss of function. These years, a growing number of researchers have been focusing on the role of intestinal flora in CNS disorders, especially the regulation over the gut-brain axis. Regulating gut microbiota with probiotics has been proposed for the prevention and treatment of various diseases, including CNS disorders [8].

The microflora in human's gastrointestinal tract is human's biggest microorganism library which consists of at least 1,000 microorganism species and has a microbial population up to 1014. Their diversity and stability vary from individual to individual and the quantity is 100 times that of human's host cells [9]. The microbiota is a dynamic ecosystem subject to multiple factors including heredity, diet, metabolism, age, geography, antibiotic therapy, and stress [10–12]. Recent evidence indicated a clear link between the change in microbiota and the cognitive behaviors [13]. In addition, some animal researches have revealed the necessity of the microbiota-gut-brain axis for the optimal function of brain activities in behavior and electrophysiology [14]. The microbiota-gut-brain axis is a bidirectional communication system that is connected by the nerve, immune, endocrine, and metabolic pathways [15]. As symbiotic bacteria, probiotics can provide potential health benefits for the host [16]. When enough probiotics are offered, they will interact actively with the endogenous microbiota. Recent studies have shown that gut microbiota plays a key role in regulating the functions of the intestinal tract and the brain. There are preliminary studies that investigated the effects of probiotics on cognitive prognosis [17]. Although a growing body of evidence suggests a close correlation between the change in intestinal flora and the development and progression of AD, no evidence says whether adding probiotics can improve cognitive impairment and pathological features of AD. As Gareau reported, intestinal imbalance in germfree animals (excluding the microbiota), enteropathogen in bacterial infection, and probiotics can regulate cognitive behaviors that include learning and memory [13].

Some complications of AD like cognitive disorder, oxidative stress, neuroinflammation, insulin resistance, and lipid metabolism are thought to be influenced by intestinal flora and probiotics. However, now there are few reports on the effects of probiotics on APP/PS1/tau triple transgenic animals. Therefore, this clinic trial aims to evaluate whether strengthening the gut microbiota with probiotic supplements can help improve AD patients' cognition and pathological changes and mitigate their neuroinflammation.

## 2. Materials and Methods

### 2.1. Experimental Animals and Grouping

In the experiment, clean grade healthy AD triple transgenic mice B6 were used; 48 129-Psen1^tm1Mpm^Tg (amyloid precursor protein [APP]Swe, tauP301L)1Lfa/J (3xTg-AD) and wt B6129SF2 mice, regardless of gender, were purchased from the Jackson Laboratory (Bar Harbor, ME, USA). The experiment was conducted in accordance with the Guide for Use of Laboratory Animals formulated by the Ethics Committee of the Second Affiliated Hospital of Qiqihar Medical University. The laboratory mice were kept in plastic cages (33 cm × 15 cm × 13 cm, *L* × *H* × W) (Makrolon, Covestro a.g., Filago, Italy) (four mice in each) at a temperature around (22 ± 1)°C and 50%–60% relative humidity in lighting conditions characterized by 12 h daylight as well as 12 h in dark (light is on at 7:00 and off at 19:00). All animals were allowed free access to water. Laboratory animals were placed in a room and separated from other animals. The experimental group and the control group were separated to avoid cross-contamination.

The 12-week-old AD mice (*n* = 24) and WT mice were divided into 2 groups, respectively: the WT + control group (*n* = 12), the WT + probiotic group (*n* = 12), the 3xTg-AD + control group (*n* = 12), and the 3xTg-AD + probiotic group (*n* = 12).

### 2.2. Probiotic Diet

The treatment started when the mice were 12 weeks old and lasted for 20 weeks. This experiment aimed at reducing the progression and functional impairment of AD. The probiotic diet-FRAMELIM® [18] (Jouxtens-Mézery, Switzerland) contains lysates of *Bifidobacterium* and *Lactobacillus acidophilus*, vitamins A and D, and w3 fatty acid from cod-liver oil, as well as vitamins B1, B3, B6, B9, and B12. It was given 5 times a week (120 mg/day) and consumed together with ordinary maintenance feed for 20 weeks. We monitored the food intake of all mice every day. The probiotic therapy would not change the animals' intake of food and water.

### 2.3. Y Maze Test

After 20 weeks' treatment, the animals underwent one-week cognitive function tests. During the test period, the animals were continuously given probiotic-supplemented diet. The Y maze (Wanlei Bio) was used to detect mice's spatial memory. Three arms are at a 120° angle from each other and each arm was 28 cm × 6 cm × 18 cm (length × width × height). Both the underside and the walls of the maze were made of white PVC. The mice were first placed at one of the arms and over the next 8 minutes, the sequence and number of their entry into the three arms were monitored [19]. An alternation is defined when a mouse visits three consecutive arms (namely, ABC, BCA, or CAB, but not CAC, BAB, or ABA). Spontaneous alternation (%) = [(number of alternations)/(total number of arms−2)] × 100.

### 2.4. Morris Water Maze (MWM)

The classical Morris water maze (MWM) experiment was conducted the day following the Y maze test. MWM is one of the classical behavioral methods used to measure spatial memory concerning brain diseases such as AD. The device is a gray round water tank with a diameter of 100 cm and a depth of 35 cm. The water there was kept at a temperature of 23 ± 2°C. The water tank was divided into four quadrants and an escape platform made of organic glass was placed 1 cm below the water surface of any of the quadrants (target quadrant). MWM consists of a 5-day place navigation test and a one-day space exploration test. During the place navigation test phase, each mouse underwent 4 tests to find the underwater platform every day. During the space exploration test phase, the underwater escape platform was removed and each mouse entered the tank randomly from two quadrants. A camera was placed at the top of the maze and connected with EthoVision software (Noldus Information Technology, Wageningen, Netherlands) to record the movement trajectory of the mouse. In each trial of the place navigation test, the mouse had 60 seconds to swim freely. If the mouse cannot find the escape platform during that period, the experimenter needs to manually guide it to the platform and let it stay 15 s. In the space exploration test, two quadrants were selected randomly to put the mice into the maze and let them swim freely in 60 s. The incubation period, swimming speed, and the swimming time in the target quadrant of each group of mice were recorded.

### 2.5. 16S rRNA Gene Sequencing for Microbiome

#### 2.5.1. Feces Collection

Feces were collected in a fume cupboard that was disinfected with ultraviolet light beforehand. Freshly collected feces were quickly put into sterile cryogenic vials and then stored in a cryogenic refrigerator.

#### 2.5.2. 16S rRNA Gene Sequencing

Samples were sent to BMKCloud (Wuhan) for detection. The detection basically consisted of the following steps: extracting total DNA from the microbiome, amplifying the target segment, recovering and purifying the amplified products, fluorescent quantitation of amplified products, and sequencing.

### 2.6. Western Blot Experiment

After all the behavioral tests were finished, the animals were anesthetized with pentobarbital sodium (50 mg/kg) before being decapitated for the brain. The hippocampi and the cortexes in the two hemispheres of the brain were separated on ice and then used for ELISA detection and the Western Blot experiment, respectively. The levels of tau (ab210703, 1 : 1000), p-tau (ab210703, 1 : 1000), GFAP (ab7260, 1 : 5000), Iba-1 (ab178846, 1 : 1000), and *ß*-actin (ab6276, 1 : 5000) (all the antibodies were from Abcam company) in the hippocampus and the cortex were determined, respectively. The secondary antibodies were from Boster (bm3895 and bm3894). The homogenates from hippocampus and cortex samples of mice were separately added along with 30 mg total DNA to 10% SDS-PAGE gel for separation. They then were electrophorized under constant voltage, transferred onto a membrane, and incubated with specific antibodies for immunoblotting assays using the ECL immunoblotting analysis system. Each gel contains molecular weight markers (10–170 kDa). The band data obtained were processed with ImageJ (NIH) and the background mean and its standard error were calculated.

### 2.7. ELISA Detection

A*β*1-40 ELISA (Invitrogen, KMB3481) and A*β*1-42 ELISA (Invitrogen, KMB3441) kits for mice were used (according to the manufacturer's instructions) to detect the concentrations of A*β*1-40 and A*β*1-42 in the hippocampus and cortex samples. A microplate reader was used to measure the optical density (OD value) at 450 nm in each well.

### 2.8. Statistical Analysis

Data are analyzed with SPSS 22.0 software. The Shapiro–Wilk test was used to evaluate the normality of data. For normally distributed data, nonparametric statistics were adopted. For duplicated data, two-way ANOVA was employed and a post hoc analysis (Bonferroni or Student–Newman–Keuls) was conducted. A *P* value <0.05 was considered statistically significant. Data are presented as mean ± SEM.

## 3. Results

### 3.1. The Probiotic-Supplemented Diet Can Alleviate the Spatial Memory Disorder of 3xTg-AD Mice

To explore the effects of the probiotic-supplemented diet on the spatial learning and memory of 3xTg-AD mice, we conducted the classical Morris water maze experiment and Y maze experiment. The Morris water maze is shown in Figure 1.  Figure 1(a) stands for the escape latency of each group of mice in the place navigation test. It can be learned from the figure that the probiotic diet did not affect the escape latency of mice in the WT group. Compared with mice in the WT + control group, those in the 3xTg-AD + control group had an obviously longer escape latency and after the probiotic dietary therapy, the escape latency of 3xTg-AD rats became remarkably shorter (*P* < 0.05).  Figure 1(b) stands for the swimming time of each group of mice in the target quadrant in the space exploration experiment. The swimming time of 3xTg-AD mice treated with the probiotic dietary therapy in the target quadrant was significantly increased (*P* < 0.05).

The spontaneous alternation accuracy of the mice in the Y maze reflected their spatial working memory. As shown in Figure 2, Figure 2(a) is the sketch map of the Y maze. It can be observed from Figure 2(b) that probiotics had no impact on the spontaneous alternation accuracy of mice in the WT group. Compared with mice in the WT + control group, those in the 3xTg-AD + control group had a lower spontaneous alternation accuracy (*P* < 0.05). After the treatment with a probiotic diet, the spontaneous alternation accuracy of mice in the 3xTg-AD + probiotic group increased (*P* < 0.05).  Figure 2(c) shows that the total number of arm entries of each group of mice in the Y maze was not statistically different (*P* > 0.05). The above result suggested that the cognitive ability of the hippocampus in 3xTg-AD mice was severely damaged. The probiotic-supplemented diet can remarkably improve the spatial memory of 3xTg-AD mice and then change their cognitive function.

### 3.2. The Probiotic-Supplemented Diet Can Improve the Pathological Features of 3xTg-AD Mice

After the end of the behavioral tests, all animals were decapitated for brains and the hippocampus and the frontal lobes were separated quickly on ice. Sandwich ELISA kit was used to detect the levels of soluble and insoluble A*β*40 and A*β*42 in the cortex and the hippocampus. As shown in Figure 3, in the 3xTg-AD + control group, the levels of soluble and insoluble A*β*40 and A*β*42 in the cortex and the hippocampus increased significantly and after probiotics were added to the diet, the levels of A*β*40 and A*β*42 declined significantly (*P* < 0.05).

The probiotic-supplemented diet can inhibit the hyperphosphorylation of tau in the cortex and hippocampus of 3xTg-AD mice. Phosphorylated Tau S202 antibodies were used for Western Blots on the cortex and hippocampus of four groups of mice. As shown in Figure 4, compared with mice in the WT + control group and the WT + probiotic group, mice in the 3xTg-AD + control group had significantly increased level of Tau S202 in the cortex and hippocampus, and mice fed a probiotic-supplemented diet in the 3xTg-AD + probiotic group had a significantly reduced level of Tau S202 in the cortex and hippocampus (*P* < 0.05).

The probiotic-supplemented diet can inhibit inflammatory responses in the brain of 3xTg-AD mice. We used specific antibodies for astrocyte and microglia to conduct Western Blot experiments on the four groups of mice, respectively. As shown in Figures 5 and 6, compared with mice in the WT + control group and the WT + probiotic group, mice in the 3xTg-AD + control group had severe inflammatory responses in the cortex and hippocampus. The mice in the 3xTg-AD + probiotic group, after the treatment with the probiotic diet, experienced reduced inflammatory responses in the cortex and hippocampus (*P* < 0.05).

### 3.3. Intestinal Flora Change in 3xTg-AD Mice

To investigate the effects of probiotics on the enteric microbiome in 3xTg-AD mice and then change their cognitive function, the fecal samples of mice were measured. The fecal specimens underwent DNA separation and species identification. According to the results, compared with mice in the WT group, those in the 3xTg-AD group exhibited a decreased diversity in intestinal flora. At the phylum level, as shown in Figure 7(a) and Table 1, compared with mice in the WT group, those in the 3xTg-AD group saw increases in the number of Helicobacteraceae, Desulfovibrionaceae, Coriobacteriaceae, Proteobacteria, Actinobacteria, and Firmicutes and a decrease in the number of Bacteroidetes. And as shown in Figure 7(b) and Table 2, at the genus level, compared with mice in the WT group, those in the 3xTg-AD group saw increases in the number of *Odoribacter*, *Helicobacter*, and *Lactobacillus* and decreases in the number of *Ruminococcus, Prevotella*, *Bacteroides*, and *Sutterella*.

## 4. Discussion

AD is a complex progressive cognitive disorder with cardinal symptoms including learning disorder, memory loss, and dysphasia [20]. Although many researches have focused on the pathogenesis of AD, the cause of AD remains unknown [21]. Probiotics are live microorganisms. Taking enough probiotics may benefit the health of the host, especially in preventing and treating AD [22]. At present, the treatment of AD can only alleviate symptoms but cannot prevent or hinder this condition. The intestinal flora plays an important role in regulating multiple neurochemical pathways of the gut-brain axis [23]; therefore, this study is focused on the intestinal flora. Probiotic therapy is becoming a recognized strategy to preventing and treating many diseases including central nervous system diseases [24] and has been proposed to be able to lower the incidence rate of AD [25]. To verify this hypothesis, we added probiotics to the diet of 3xTg-AD mice, further observed changes in cognitive behaviors and pathological feature of AD, and explored the change in intestinal flora of 3xTg-AD mice and WT mice. This study can help offer new strategies for treating AD.

In this study, APP/PS1/tau triple transgenic (3xTg) mice with overexpressed mutants APP (APPSWE), PS1 (PS1M146V), and tau (tauP301L) were used to investigate the effects of a probiotic diet on 3xTg-AD. The research results showed that, compared with mice in the WT group, those in the 3xTg-AD group had a damaged spatial memory, increased levels of soluble and insoluble A*β*40 and A*β*42 in the hippocampus and cortex, and neurofibrillary tangles and inflammatory reactions. However, when given a probiotic diet, the above symptoms of the 3xTg-AD mice were mitigated.

To verify this hypothesis, 3xTg-AD mice underwent the probiotic-supplemented dietary therapy. The Morris water maze experiment showed that the probiotic diet can mitigate the damage of learning memory of 3xTg-AD mice. In the Y maze experiment, probiotics did not impact the spontaneous alternation accuracy of mice in the WT group, but improved the spontaneous alternation accuracy of 3xTg-AD mice. However, this did not influence the total number of arm entries of mice in each group, indicating that the probiotic-supplemented diet can significantly improve 3xTg-AD mice's spatial memory and then change their cognitive function. Bonfili et al. [26] proved that the daily oral administration of probiotics reversed the damage of working memory on APP/PS1 mice in the Y maze. The study by Savignac et al. showed that taking probiotics for a long time can improve APP/PS1 mice's ability to identify new objects and their learning and memory in the Barnes maze [27]. The latest randomized double-blind controlled clinical trial demonstrated that giving a mixture of probiotics for 12 weeks could have positive effects on AD patients' cognitive function and certain metabolic status [28]. According to the research result of Elmira Akbari, AD patients treated with probiotics showed some improvement in MMSE scores [29].

It is known that reducing or eliminating the production of A*β* is an important strategy for the treatment of Alzheimer's disease [30]. According to research reports, one of the hallmark neuropathological features of AD is the senile plaques, a result of the accumulation of A*β* [31]. Since 3xTg-AD mice present senile plaques normally when they are 12 months old, we detected the levels of A*β*40 and A*β*42 in the hippocampus and the cortex separately with ELISA [32]. It was reported that A*β*40 and A*β*42 are neurotoxic peptides generated from proteolysis of APP by *ß*-secretase and *γ*-secretase [33, 34] successively. On the contrary, *α*-secretase (a disintegrin and metalloprotease 10, ADAM10) disintegrates APP in the final A*β* sequence and hinders the production of A*β* [35]. In addition, A*β* can be degraded and eliminated by IDE and NEP. Maintaining a balance between the production and elimination of A*β* is considered a potential strategy for treatment [36]. A*β* comes in many forms and A*β*40 and A*β*42 are the most abundant forms in the brain. Its abnormal deposition will affect the normal activity of neurons and jeopardize the homeostasis of the neural network. The result of this study showed that giving a probiotic-supplemented diet to 3xTg-AD mice for 20 weeks can downregulate the levels of soluble and insoluble A*β*40 and A*β*42 in the hippocampus and cortex.

Neurofibrillary tangles, the aggregates of hyperphosphorylated tau protein, are another neuropathological feature of AD. The pathological development of tau is linked with progressive neuronal loss and memory dysfunction [37]. In the progression of AD, tau is hyperphosphorylated at S202. Hindering the hyperphosphorylation of tau protein has become a hot button in the current drug research for AD. The pathological formation of tau protein can cause turbulence in microtubules, making them unstable and damaging their key function in axonal transport, and resulting in synaptic dysfunction and neuronal degeneration [38, 39]. Our research result indicated that, in the cerebral cortex and hippocampus of 3xTg mice, the probiotic diet reduced the increase in phosphorylation of tau at S201.

Neuroinflammation is also a vital pathological hallmark of AD and is mediated by activated microglia and reactive astrocyte, with Ib*α*1 and GFAP as the markers, respectively [40]. Some studies have shown that A*β* can induce oxidative stress in mice's brains, activate microglia and astrocyte, and cause neuroinflammation, neuronal damage, and cognitive disorder [41]. As expected, we also found that the probiotic diet is a strong neuroprotective agent that can protect the neurons of 3xTg-AD mice from the erosion of neuroinflammation.

In recent years, a growing number of studies have reported that there exists a close link between intestinal flora and nerve system diseases and it is called the gut-brain axis. The intestinal flora of an AD patient is vastly different from that of a normal person in composition, which indicates that the AD patient's composition of intestinal flora may be involved in the development of a*β* amyloidosis in the brain.

## 5. Conclusion

In order to explore the change in and composition of the intestinal flora of the 3xTg-AD group, we determined the bacterial community in the fecal specimen with the 16S rRNA sequencing technique. The detection results showed a decreased *α*-diversity, a total statistical index of 3xTg-AD mice. Compared with mice in the WT group, those in the 3xTg-AD group had seen increases in the number of Helicobacteraceae, Desulfovibrionaceae, Coriobacteriaceae, Actinobacteria, and Firmicutes and a decrease in the number of Bacteroidetes; and increases in the number of Odoribacter, Helicobacter, and Lactobacillus and a decrease in the number of Prevotella. Those changes were consistent with what have been discovered in AD patients [42]. The change in intestinal flora may be linked with the cognitive impairment, pathological manifestations, and inflammatory responses observed in 3xTg-AD mice. It is worthy of further study.

In a word, the probiotic-supplemented diet can improve 3xTg-AD model mice's cognitive function and reverse pathological manifestations of AD and the pathological changes of AD and the cognitive disorder are linked with the change in intestinal flora. The study reinforces the idea that the probiotic therapy can prevent and treat AD and is worthy of future investigation.

## Figures and Tables

**Figure 1:** The probiotic-supplemented diet can improve the spatial and learning memory of 3xTg-AD mice. Morris water maze experiment. (a) Escape latency of each group of mice. (b) Swimming time of each group of mice in the target quadrant. ^*∗*^*P* < 0.05; ^*∗∗*^*P* < 0.01.

**Figure 2:** The probiotic-supplemented diet can improve the spatial working memory of 3xTg-AD mice. (a) Sketch map of the Y maze experiment. (b) Histogram of Y maze spontaneous alternation accuracy. (c) Histogram of total number of arm entries in the Y maze (*P* > 0.05); ^*∗*^*P* < 0.05.

**Figure 3:** The probiotic-supplemented diet can lower the levels of A*β*40 and A*β*42 in the cortex and hippocampus of 3xTg-AD mice. (a) Histogram of soluble A*β*40 in the cortex of four groups of mice. (b) Histogram of soluble A*β*40 in the hippocampus of four groups of mice. (c) Histogram of soluble A*β*42 in the cortex of four groups of mice. (d) Histogram of soluble A*β*42 in the hippocampus of four groups of mice. (e) Histogram of insoluble A*β*40 in the cortex of four groups of mice. (f) Histogram of insoluble A*β*40 in the hippocampus of four groups of mice. (g) Histogram of insoluble A*β*42 in the cortex of four groups of mice. (h) Histogram of insoluble A*β*42 in the hippocampus of four groups of mice. ^*∗*^*P* < 0.05; ^*∗∗*^*P* < 0.01; ^*∗∗∗*^*P* < 0.001.

**Figure 4:** The probiotic-supplemented diet can lower the levels of p-tau in the cortex and hippocampus of 3xTg-AD mice. Histogram of p-tau level in the (a) cortex and (b) hippocampus of four groups of mice; ^*∗∗*^*P* < 0.01.

**Figure 5:** The probiotic-supplemented diet can lower the GFAP level in the cortex and hippocampus of 3xTg-AD mice. Histogram of GFAP level in the (a) cortex and (b) hippocampus of four groups of mice. ^*∗*^*P* < 0.05; ^*∗∗*^*P* < 0.01.

**Figure 6:** The probiotic-supplemented diet can lower the Iba-1 level in the cortex and hippocampus of 3xTg-AD mice. Histogram of Iba-1 level in the (a) cortex and (b) hippocampus of four groups of mice. ^*∗*^*P* < 0.05; ^*∗∗*^*P* < 0.01.

**Figure 7:** Changes in the intestinal flora of 3xTg-AD mice. Flora distribution of WT mice and 3xTg-AD mice at the (a) phylum level and (b) genus level.

**Table 1:** Data of Figure 7(a).

	Helicobacteraceae (%)	Desulfovibrionaceae (%)	Coriobacteriaceae (%)	Proteobacteria (%)	Actinobacteria (%)	Fusobacteria (%)	Verrucomicrobia (%)	Firmicutes (%)	Bacteroidetes (%)	Others (%)
WT	0.01	0.05	0.02	0.002	0.01	0.001	0.001	0.5	0.22	0.31
3xTg-AD	0.15	0.15	0.19	0.04	0.1	0.002	0.001	0.15	0.35	0.01

**Table 2:** Data of Figure 7(b).

	*Odoribacter*b (%)	*Helicobacter* (%)	*Ruminococcus* (%)	*Prevotella* (%)	*Bacteroides* (%)	*Sutterella* (%)	*Lactobacillus* (%)	Others (%)
WT	0.001	0.07	0.045	0.6	0.026	0.04	0.04	0.178
3xTg-AD	0.3	0.31	0.02	0.001	0.002	0	0.32	0.047

## Data Availability

The datasets used and/or analyzed during the present study are available from the corresponding author on reasonable request.
